# MiR-362-3p functions as a tumor suppressor through targeting MCM5 in cervical adenocarcinoma

**DOI:** 10.1042/BSR20180668

**Published:** 2018-06-21

**Authors:** Dan Wang, Hongyan Wang, Yichun Li, Qian Li

**Affiliations:** 1 Department of Gynecology, Jining No.1 People’s Hospital, Jining 272000, Shandong, China; 2 Department of Hepatobiliary Surgery, Jining No.1 People’s Hospital, Jining 272000, Shandong, China

**Keywords:** biomarker, cervical cancer, microRNA, miR-362-3p, MCM5

## Abstract

Our previous study suggested that minichromosome maintenance protein 5 (MCM5) overexpression was observed in cervical adenocarcinoma and closely associated with advanced clinical stage, more metastatic lymph nodes, present distant metastasis, low histological grade, and poor prognosis. Down-regulation of MCM5 inhibited cervical adenocarcinoma cell proliferation. The purpose of the present study is to search and confirm valuable microRNAs (miRNAs), which target MCM5 to modulate cervical adenocarcinoma cell proliferation. In our results, we found that levels of miR-362-3p expression were reduced in cervical adenocarcinoma tissues and cell lines. Moreover, 3′-UTR of MCM5 had binding site of miR-362-3p through analyzing Targetscan database and miRanda database, and there were an inverse association between miR-362-3p and MCM5 in cervical adenocarcinoma tissues. Furthermore, we verified miR-362-3p directly targeted to 3′-UTR of DCLK1 by luciferase reporter assay, and negatively regulated mRNA and protein expressions of MCM5 by qPCR and Western blot. Then, we conducted gain-of-function study and rescued-function study, and found that miR-362-3p served as a tumor suppressive miRNA to modulate cervical adenocarcinoma cell proliferation through regulating the functional target MCM5. Finally, we analyzed correlations between miR-362-3p expression and clinicopathological characteristics and observed that miR-362-3p low expression was associated with advanced clinical stage and poor prognosis. In conclusion, miR-362-3p is a tumor suppressive miRNA in cervical adenocarcinoma.

## Introduction

Cervical cancer is one of the most common gynecologic cancers worldwide with an estimated 527,600 cases and 254,700 deaths according to the GLOBOCAN 2012 data [1]. The increasing trend of incidence and mortality of cervical cancer was observed in Chinese Cancer Statistics, which reported that there are approximately 98,900 new cervical cancer cases and 30,500 deaths due to cervical cancer in 2015 [2]. Cervical adenocarcinoma accounts for 20–25% of all cervical cancer cases [3]. Due to aggressive phenotype and radiotherapy resistance, the prognosis of cervical adenocarcinoma is unsatisfactory [4]. Our previous study suggested that minichromosome maintenance protein 5 (MCM5) overexpression was observed in cervical adenocarcinoma and closely associated with advanced clinical stage, more metastatic lymph nodes, present distant metastasis, low histological grade, and poor prognosis [5]. Moreover, the experiments *in vitro* indicated that down-regulation of MCM5 inhibited the proliferation of Hela and GH354 cells [5]. MCM5 may serve as a potential therapeutic target for cervical adenocarcinoma.

In the past decades, microRNAs (miRNAs) have been showed to be involved in human carcinogenesis [6–8]. In neuroblastoma, MCM5 was a functional target for miR-885-5p to inhibit tumor cells proliferation and survival [9]. In our early study, we observed miRNA target databases and found miR-362-3p target sequences of the MCM5 3′-UTR. Moreover, miR-362-3p has been found to function as a tumor suppressor in most types of human cancer [10,11]. Meanwhile, we conducted correlation analysis between miRNAs and MCM5 in cervical adenocarcinoma and found that MCM5 expression was negatively correlated with the miR-362-3p expression, but had no association with the miR-885-5p. Therefore, the aim of our study is to confirm the correlation between miR-362-3p and MCM5 in cervical adenocarcinoma, and investigate the role of miR-362-3p in cervical adenocarcinoma.

## Materials and methods

### Sample collection

For the use of these clinical materials for research purposes, prior written informed consent from all the patients and approval from the Ethics Committees of Jining No.1 People’s Hospital were obtained. A total of 78 fresh cervical adenocarcinoma tissue specimens and 20 fresh normal cervical tissue specimens were obtained from Jining No.1 People’s Hospital (Shandong, China). Clinical samples were collected at the time of diagnosis before any therapy. All specimens had confirmed pathological diagnosis by two pathologists.

### RNA extraction and quantitative RT-PCR (qPCR)

RNA isolation (RNAiso Plus, Takara, Japan) and MCM5 mRNA expression determination were carried out according to previous description [5]. The sequence-specific forward and reverse primers sequences for MCM5 were 5′-AGCATTCGTAGCCTGAAGTCG-3′ and 5′-CGGCACTGGATAGAGATGCG-3′ respectively. Forward and reverse primer sequences for GAPDH mRNA were 5′-GGAGCGAGATCCCTCCAAAAT-3′ and 5′-GGCTGTTGTCATACTTCTCATGG-3′ respectively. The isolated total RNA was reverse transcribed using the One Step PrimeScript miRNA cDNA Synthesis Kit (Takara, Japan) for miR-362-3p, according to the manufacturer’s instructions. The sequence-specific forward primers for mature miR-362-3p, U6 internal control, and the Uni-miR qPCR Primer were purchased from Takara. The reactions were performed using SYBR Premix Ex TaqTM II (Takara, Japan) on a Light Cycler (Roche Diagnostics, U.S.A.). Relative expression of miR-362-3p was calculated via the comparative cycle threshold method and normalized to the expression of U6.

### Immunohistochemistry

Immunohistochemical analysis was performed to measure MCM5 protein expression in cervical adenocarcinoma tissue samples according to previous description [5].

### The Cancer Genome Atlas database analysis

The Cancer Genome Atlas database was used to analyze the prognostic significance of miR-362-3p in cervical cancer patients. The cervical cancer patient’s cohort from Cancer Genome Atlas database included 264 cases.

### Western blot

Western blot analysis was performed according to previous description [5]. The target protein antibodies included MCM5 (1:1000 dilution, Abcam, U.S.A.) and β-actin (1:3000 dilution, Santa Cruz, U.S.A.). Quantity One Software (Bio-Rad, U.S.A.) was used to analyze the intensity of the blots.

### Cell lines culture and cell transfection

The cell culture of Ect1/E6E7, End1/E6E7, Hela and GH354, and cell transfection of siRNA/pcDNA were carried out according to previous description [5]. The mimics-miR-363-3p, mimics-NC, inhibitor-miR-363-3p, and inhibitor-NC were purchased from RiboBio (Guangzhou, China) and used at 20 mM Opti-MEM transfection media, and lipofectamine 2000 (both from Invitrogen, U.S.A.) was used to transfect the cells once they reached 60% confluency. The qPCR was used to test the transfection efficiencies of mimics-miR-363-3p and inhibitor-miR-363-3p in Hela and GH354 cells.

### Bioinformatics analysis and luciferase reporter assay

Targetscan database and miRanda database were used to analyze the putative target genes of miR-362-3p. The MCM5 wild-type (wt) and mutant (mut) 3′-UTR were created and cloned to the firefly luciferase-expressing vector, the pmiR-RB-REPORT luciferase reporter plasmid (RiboBio, China). For the luciferase assay, Hela and GH354 cells were seeded in 24-well plates and cotransfected with the pmiR-MCM5-wt/pmiR-MCM5-mut and mimics-miR-363-3p/inhibitor-miR-363-3p by using lipofectamine 3000 (Invitrogen, U.S.A.). Luciferase activities were determined with the Dual-Luciferase Reporter System (Promega, U.S.A.).

### Cell proliferation assays

Cell proliferation was analyzed using 3-(4,5-cimethylthiazol-2-yl)-2,5-diphenyl tetra-zolium bromide (MTT, Sigma, U.S.A.) assay and colony formation assay according to previous description [5]. After transfection, cells were grown in a 96-well plate for 24, 48, 72, and 96 h, and in a six-well plate for 12 days.

### Statistical analysis

SPSS 13.0 software (SPSS, U.S.A.) and GraphPad Prism 5.0 (GraphPad Software Inc., U.S.A.) software were used for statistical analysis. The differential of miR-362-3p expression between cervical adenocarcinoma tissue specimens and normal cervical tissue specimens was analyzed by Wilcoxon signed rank test. The Student’s *t*-test was used for comparisons of two independent groups. One-way analysis of variance was used to analyze the differences among more than two groups. The χ^2^ test was employed to analyze the association between miR-362-3p expression and clinicopathological characteristics in cervical adenocarcinoma patients. Kaplan–Meier method was used to conduct the survival analysis. The univariate and multivariate cox regression analyses were used to evaluate the prognostic significance of miR-362-3p in cervical adenocarcinoma. The Spearman test was applied to explore the correlation between MCM5 expression and miR-362-3p expression. All assays were independently repeated three times. A *P*-value of less than 0.05 was considered statistically significant.

## Results

### MiR-362-3p expression is decreased in cervical adenocarcinoma

In order to explore the expression of miR-362-3p in cervical adenocarcinoma, qPCR was executed to detect miR-362-3p in cervical adenocarcinoma tissues, normal cervical tissues, normal ectocervical cell line (End1/E6E7), normal endocervical cell line (End1/E6E7), and two cervical adenocarcinoma cell lines (Hela and GH354). The expression of miR-362-3p was decreased in cervical adenocarcinoma tissues compared with normal cervical tissues (*P*<0.001, Figure 1A). Meanwhile, miR-362-3p expression levels were reduced in cervical adenocarcinoma cell lines (Hela and GH354) compared with normal cervical cell lines (End1/E6E7 and End1/E6E7) (*P*<0.001, Figure 1B).

**Figure 1:** The expression of miR-362-3p in cervical adenocarcinoma tissue and cell (**A**) MiR-362-3p expression is reduced in cervical adenocarcinoma tissue compared with normal cervical tissues. (**B**) Levels of miR-362-3p expression are reduced in cervical adenocarcinoma cell lines (Hela and GH354) compared with normal cervical cell lines (End1/E6E7 and End1/E6E7). (**C**) The efficiencies of miR-362-3p mimics and miR-362-3p inhibitor are confirmed by qPCR.

In order to study the biological functions of miR-362-3p in cervical adenocarcinoma, we performed loss-of-function study and gain-of-function study in cervical adenocarcinoma cell lines. We induced up-regulation of miR-362-3p in Hela by mimics-miR-362-3p and down-regulation of miR-362-3p in GH354 by inhibitor-miR-362-3p, and these efficiencies were confirmed by qPCR (Figure 1C).

### MiR-362-3p binds to the 3′-UTR of MCM5 and regulates MCM5 expression

According to miRNA target databases and published studies, we found that miR-362-3p may directly target the 3′-UTR of MCM5. The predicted binding site of miR-362-3p on MCM5 3′-UTR was suggested in Figure 2A. We further explored the association between miR-362-3p and MCM5 mRNA expression in cervical adenocarcinoma tissues by qPCR and found that miR-362-3p was oppositely associated with MCM5 mRNA expression in cervical adenocarcinoma tissues (*r* = −0.720, *P*<0.001, Figure 2B). Moreover, we analyzed the association between miR-362-3p and MCM5 protein expression in cervical adenocarcinoma tissues by qPCR and immunohistochemistry, and also found a negative correlation between miR-362-3p and MCM5 protein expression (r = −0.748, *P*<0.004, Table 1). Furthermore, we performed luciferase reporter assay to confirm the predicted binding site miR-362-3p on MCM5 3′-UTR, and found mimics-miR-362-3p obviously down-regulated the luciferase activity of the pmiR-MCM5-wt in the Hela cell (Figure 4C, *P*<0.001) and inhibitor-miR-362-3p markedly up-regulated the luciferase activity of the pmiR-MCM5-wt (*P*<0.001, Figure 2C). Furthermore, we found that mimics-miR-362-3p significantly suppressed mRNA and protein expressions of MCM5, and inhibitor-miR-362-3p significantly elevated mRNA and protein expressions of MCM5 (Figure 2D,E). These data proved that miR-362-3p negatively regulates MCM5 mRNA and protein expression through directly targeting its 3′-UTR.

**Figure 2:** The relationship between miR-362-3p and MCM5 in cervical adenocarcinoma (**A**) Position of the miR-362-3p target site in 3′-UTR of MCM5 mRNA. (**B**) An inverse correlation between miR-362-3p and MCM5 expression in the same set of cervical adenocarcinoma. (**C**) Relative luciferase activity of Hela and GH354 cells after cotransfection with pmiR-MCM5-wt or pmiR-MCM5-mut, and miR-362-3p mimics or miR-362-3p inhibitor. (**D** and **E**) MCM5 mRNA and protein expressions are detected after miR-362-3p mimics transfected in Hela and miR-362-3p inhibitor transfected in GH354 by qPCR and Western blot.

**Table 1:** The association between miR-362-3p and MCM5 protein in cervical adenocarcinoma

Group		miR-362-3p		*r*	*P*
		High expression	Low expression		
MCM5 protein	High expression	7	36	-0.748	<0.001
	Low expression	32	3		

### MCM5 is a functional target of miR-362-3p to modulate cervical adenocarcinoma cell proliferation

We investigated the effect of miR-362-3p on the proliferation of cervical adenocarcinoma cells through MTT assay and colony formation assay. The growth curves determined by MTT assay indicated that up-regulation of miR-362-3p significantly suppressed Hela cell proliferation, and down-regulation of miR-362-3p significantly promoted GH354 cell proliferation (both *P*<0.05, Figure 3A). The colony formation assay showed that up-regulation of miR-362-3p obviously reduced the number of colonies in Hela cell line, and down-regulation of miR-362-3p obviously elevated the number of colonies in GH354 cell line (both *P*<0.05, Figure 3B).

**Figure 3:** MCM5 is a functional target of miR-362-3p to modulate cervical adenocarcinoma cell proliferation Transfection with miR-362-3p mimics suppresses Hela cell proliferation, and transfection with miR-362-3p inhibitor accelerates GH354 cell proliferation (**A** and **B**). Cotransfection of miR-362-3p mimics and pcDNA-MCM5 rescues inhibition of miR-362-3p mimics in Hela cell proliferation (A and B). Cotransfection of miR-362-3p inhibitor and siRNA-MCM5 reversed facilitation of miR-362-3p inhibitor in GH354 cell (A and B).

The inhibition of down-regulating MCM5 on cervical adenocarcinoma cell proliferation has been proved in our previous study [5]. The above results suggested that miR-362-3p negatively regulates MCM5 expression through binding to the 3′-UTR of MCM5. Therefore, we supposed that MCM5 is a functional target of miR-362-3p to modulate cervical adenocarcinoma cell proliferation. In order to confirm our guess, we conducted rescued-function studies through cotransfecting mimics-miR-362-3p and pcDNA-MCM5 into Hela cells, and inhibitor-miR-362-3p and siRNA-MCM5 into GH354 cells. We found that cotransfection of mimics-miR-362-3p and pcDNA-MCM5 markedly rescued inhibition of miR-362-3p in Hela cell proliferation (both *P*<0.05, Figure 3A), and cotransfection of inhibitor-miR-362-3p and siRNA-MCM5 markedly rescued facilitation of inhibitor-miR-362-3p in GH354 cell proliferation (both *P*<0.05, Figure 3B). Thus, MCM5 is a functional target of miR-362-3p involving in cervical adenocarcinoma cell proliferation.

### MiR-362-3p low expression is associated with clinical stage of cervical adenocarcinoma patients

In order to further assess the clinical value of miR-362-3p in cervical adenocarcinoma patients, we observed correlations between miR-362-3p expression and clinicopathological characteristics in 78 cervical adenocarcinoma cases. All cervical adenocarcinoma patient cases were divided into miR-362-3p low-expression group and miR-362-3p high-expression group based on the median expression level [12,13]. The relationship between clinicopathological characteristics and miR-362-3p expression was showed in Table 2. There was no significant association of miR-362-3p expression with patients’ age (*P*=0.495), tumor size (*P*=0.819), lymph node metastasis (*P*=0.174), distant metastasis (*P*=0.482), histological grade (*P*=0.105), and HPV infection (*P*=0.111). However, the miR-362-3p expression was closely correlated with clinical stage (I–IIA vs IIB–IV, *P*=0.035).

**Table 2:** Association between miR-362-3p expression and clinicopathological characteristics in cervical adenocarcinoma patients

Characteristics	*n*	miR-362-3p expression		*P*
		High (%)	Low (%)	
Age (y)				
≤50	35	16 (45.7)	19 (54.3)	0.495
>50	43	23 (53.5)	20 (46.5)	
Clinical stage				
I–IIA	29	19 (65.5)	10 (34.5)	0.035
IIB–IV	49	20 (40.8)	29 (59.2)	
Tumor size (cm)				
≤4	45	23 (51.1)	22 (48.9)	0.819
>4	33	16 (48.5)	17 (51.5)	
Lymph node metastasis				
Absent	40	23 (57.5)	17 (42.5)	0.174
Present	38	16 (42.1)	22 (57.9)	
Distant metastasis				
Absent	71	37 (52.1)	34 (47.9)	0.428
Present	7	2 (28.6)	5 (71.4)	
HPV				
Absent	43	18 (41.9)	25 (58.1)	0.111
Present	35	21 (60.0)	14 (40.0)	
Histological grade				
Well	31	19 (61.3)	12 (38.7)	0.105
Moderately/Poorly	47	20 (42.6)	27 (57.4)	

### MiR-362-3p low expression is associated with poor prognosis of cervical adenocarcinoma patients

In order to investigate the prognostic value of miR-362-3p expression for cervical cancer patients, we dissected cervical cancer patient cohort including 264 cases from The Cancer Genome Atlas database and found that miR-362-3p low expression had shorter overall survival time than those with miR-362-3 high expression (*P*=0.003, Figure 4A). Furthermore, Kaplan–Meier analysis and log-rank test were used to assess the correlation between the miR-362-3p and cervical adenocarcinoma patients’ overall survival. In 78 cervical adenocarcinoma patients with prognosis information, we observed that expression level of miR-362-3p was obviously correlated with cervical adenocarcinoma patients’ overall survival, as cervical adenocarcinoma patients with high expression of miR-362-3p had better survival than those with low expression of miR-362-3p (*P*=0.011, Figure 4B). Univariate and multivariate analyses of overall survival duration in cervical adenocarcinoma patients have been showed in a previous study. In the present study, we further analyzed the prognostic value of miR-362-3p in cervical adenocarcinoma patients and found that high expression of miR-362-3p is an favorable prognostic factor for cervical adenocarcinoma patients based on univariate analysis (HR, 95% CI: 0.473, 0.261–0.8569; *P*=0.013, Table 3), but not an independent prognostic factor multivariate analysis (HR, 95% CI: 0.633, 0.334–1.201; *P*=0.162, Table 3).

**Figure 4:** The prognostic significance of miR-362-3p in cervical adenocarcinoma (**A**) Cervical adenocarcinoma patients with miR-362-3p low expression have shorter overall survival time than those with miR-362-3 high expression based on Cancer Genome Atlas database. (**B**) MiR-362-3p expression is positively correlated with overall survival in cervical adenocarcinoma patients based on our study.

**Table 3:** Summary of univariate and multivariate Cox regression analysis of overall survival duration in cervical adenocarcinoma patients

Parameter	Univariate analysis			Multivariate analysis		
	*P*	HR	95% CI	*P*	HR	95%CI
MiR-362-3p expression (low vs high)	0.013	0.473	0.261–0.856	0.162	0.633	0.334–1.201

95% CI, 95% confidence interval; HR, hazard ratio; Multivariate analysis is adjusted to clinical stage, lymph node metastasis, distant metastasis, HPV, and histological grade.

## Discussion

The status of MCM5 mRNA and protein has been found overexpressed in cervical adenocarcinoma tissues and cell lines in our previous study [5]. Meanwhile, MCM5 high expression was correlated with advanced clinical stage, more lymph node metastasis, present distant metastasis, low histological grade, and poor prognosis, and down-regulation of MCM5 expression inhibited cervical adenocarcinoma cell proliferation *in vitro* [5]. The purpose of the present study is to search and confirm valuable miRNAs, which target MCM5 to modulate cervical adenocarcinoma cell proliferation. Afanasyeva et al. [9] reported that miR-885-5p has a tumor suppressive role in regulating neuroblastoma cell cycle progression and cell survival through binding 3′- UTR of MCM5. In our early study, we found that there was no association between miR-885-5p and MCM5 in cervical adenocarcinoma tissues. Fortunately, we found that the 3′-UTR of MCM5 had binding site of miR-362-3p through analyzing Targetscan database and miRanda database, and there was an inverse association between miR-362-3p and MCM5 in cervical adenocarcinoma tissues. These evidences implied that MCM5 is a target of miR-362-3p. In order to confirm the relationship between miR-362-3p and MCM5, the luciferase reporter assay, qPCR and Western blot were performed in cervical adenocarcinoma cells. We found that miR-362-3p negatively regulates MCM5 mRNA and protein expression through directly targeting its 3′-UTR.

The biological function of miR-362 has been explored in several types of human cancers. Wu et al. [14] indicated that miR-362-5p inhibited neuroblastoma cell growth, migration, and invasion partially through targeting phosphatidylinositol 3-kinase-C2β. Moreover, Christensen et al. [15] demonstrated that miR-362-3p reduced cell viability and induced cell cycle arrest via regulating target genes including E2F1, USF2, and PTPN1 in colorectal cancer. In cervical cancer, miR-362-5p has been suggested to function as an antioncogenic miRNA to regulate cell proliferation, migration, and invasion through targeting SIX1 [16]. The biological function of miR-362-3p in cervical adenocarcinoma was still unknown. We conducted gain-of-function study and rescued-function study and found that miR-362-3p served as a tumor suppressive miRNA to modulate cervical adenocarcinoma cell proliferation through regulating the functional target MCM5.

The status of miR-362 expression has been shown dysregulated in several types of human malignancies, which has high expression or low expression in cancer tissues depending on the tumor type. The expression of miR-362 suggested decrease in neuroblastoma [14], colorectal cancer [15,17], cervical cancer [16], breast cancer [18], renal cancer [19] and astrocytoma [20], and increased in hepatocellular carcinoma [21,22], chronic myelocytic leukemia [23], breast cancer [21], renal cancer [24], and gastric cancer [25,26]. Interesting results were observed in breast cancer and renal cancer, miR-362-3p expression was elevated in tumor tissues, and miR-362-5p expression was reduced in tumor tissues [18,19,21,24]. In cervical cancer, Shi et al. [16] showed that miR-362-5p was decreased in tumor tissues and cell lines. Similarly, we also found that miR-362-3p expression decreased in cervical adenocarcinoma tissues and cell lines compared with normal cervical tissues and normal cervical cell lines respectively. Furthermore, we analyzed correlations between miR-362-3p expression and clinicopathological characteristics and found that the miR-362-3p expression was negatively correlated with clinical stage in cervical adenocarcinoma patients. Shi et al. [16] also suggested that low expression of miR-362-5p was associated with FIGO stage, lymph node metastasis, and vascular invasion in cervical cancer. In neuroblastoma patients, miR-362-5p expression was associated with neuroblastoma risk factors such as young age, advanced stage, and strong metastasis potential [14]. However, Zhang et al. [26] indicated that miR-362-3p high expression was correlated with deeper local invasion and diffuse type in gastric cancer patients.

The present results indicated a lack of prognostic significance of miR-362-3p in cervical cancer, even though earlier studies reported the prognostic value in breast cancer [18] and colorectal cancer [15]. In breast cancer, Kang et al. [18] demonstrated that there was no significant correlation between miR-362-3p expression and relative survival duration. Christensen [15] revealed that colorectal cancer patients with no recurrence had a higher level of miR-362-3p expression compared with recurrent patients, and there was an obviously positively correlation between miR-362-3p expression and disease-free survival in colorectal cancer. In order to assess the prognostic value of miR-362-3p in cervical adenocarcinoma patients, we first analyzed the Cancer Genome Atlas database and found that miR-362-3p low expression had shorter overall survival time that those with miR-362-3 high expression. Furthermore, low expression of miR-362-3p is an unfavorable prognostic factor, but not an independent prognostic factor for cervical adenocarcinoma patients. Due to the limited sample size in the present study, more studies would be needed to further confirm the prognostic significance of miR-362-3p in cervical adenocarcinoma patients.

In conclusion, miR-362-3p is a tumor suppressive miRNA to modulating cervical adenocarcinoma cell proliferation through binding to the functional target MCM5. The low expression of miR-362-3p is associated with advanced clinical stage and poor prognosis.

## Abbreviations

HPV: human papillomavirus
MCM5: minichromosome maintenance protein 5
miRNA: microRNA
mut: mutant
wt: wild-type
